# Human Posture Detection Method Based on Wearable Devices

**DOI:** 10.1155/2021/8879061

**Published:** 2021-03-24

**Authors:** Xiaoou Li, Zhiyong Zhou, Jiajia Wu, Yichao Xiong

**Affiliations:** ^1^College of Medical Instruments, Shanghai University of Medicine & Health Sciences, Shanghai 201318, China; ^2^School of Design and Art, Shanghai Dianji University, Shanghai 200240, China

## Abstract

The dynamic detection of human motion is important, which is widely applied in the fields of motion state capture and rehabilitation engineering. In this study, based on multimodal information of surface electromyography (sEMG) signals of upper limb and triaxial acceleration and plantar pressure signals of lower limb, the effective virtual driving control and gait recognition methods were proposed. The effective way of wearable human posture detection was also constructed. Firstly, the moving average window and threshold comparison were used to segment the sEMG signals of the upper limb. The standard deviation and singular values of wavelet coefficients were extracted as the features. After the training and classification by optimized support vector machine (SVM) algorithm, the real-time detection and analysis of three virtual driving actions were performed. The average identification accuracy was 90.90%. Secondly, the mean, standard deviation, variance, and wavelet energy spectrum of triaxial acceleration were extracted, and these parameters were combined with plantar pressure as the gait features. The optimized SVM was selected for the gait identification, and the average accuracy was 90.48%. The experimental results showed that, through different combinations of wearable sensors on the upper and lower limbs, the motion posture information could be dynamically detected, which could be used in the design of virtual rehabilitation system and walking auxiliary system.

## 1. Introduction

A human posture detection system means identifying the change of posture in a specified area and detecting the range of human motion. Generally, it can be described quantitatively by the devices. According to different detection approaches, the human posture detection is mainly divided into nonwearable detection and wearable detection. In the meantime, there are four kinds of human posture detection modes, that is, infrared detection, data clothing and data gloves, electronic camera, and measurement sensors. For the wearable detection combined with the measurement sensors, there are several characteristics of small detection limit and no interference from external environment such as background illumination.

Surface electromyography (sEMG) represents the bioelectrical activities of spinal cord motor neurons under the control of cerebral motor cortex, which can directly reflect the human motion intention and muscle state information with real-time interaction and noninvasive and convenient operation [1]. A novel muscle-computer interface (MCI) based on the sEMG signal features has been proposed, which can be used to identify limb motion patterns and convert them into input commands to control external devices. This technology has been applied in the field of rehabilitation; for example, it can help patients with the motor dysfunction perform motor control in a virtual reality (VR) environment and effectively improve the effect of rehabilitation training [2, 3]. Rincon et al. designed an immersive rehabilitation video game, which used Unity Engine and sEMG sensors to capture the movement action [4]. Powell et al. used the VR environment to perform myoelectricity control training based on pattern recognition, which improved the consistency and discrimination of myoelectricity signals of stump muscles in amputees [5]. The introduction of the sEMG signal analysis implements intelligent confirmation of system instructions, which can solve the problem of limb dyskinesia.

The gait is the posture performance of human walking, which reflects the structure and function of human motion and nervous system. The purpose of gait detection is to identify the gait patterns of subjects by analyzing their gait information. The main ways of information acquisition include acceleration sensor, pressure sensor, and multisensor fusion [6–9]. Young and Omid used the machine learning method to process the gait information of acceleration sensor and obtained higher classification accuracy [10, 11]. The gait detection based on multisensor fusion can obtain more gait information, which is helpful in improving the identification accuracy. The gait detection technology has been widely used in sport training, medical research, and pedestrian navigation [12–14].

In this study, an effective method of wearable human posture detection on upper and lower limbs was proposed. The sEMG signal analysis of upper limb was applied to virtual driving. Based on the characteristics of real-time and safety of the sEMG signal, the virtual driving operation was performed by effective feature extraction and classification identification. By combining the features of triaxial acceleration and plantar pressure, an optimized support vector machine (SVM) classifier was used to obtain the effective results of gait identification.

## 2. Methods

The gesture and gait movements are important body language. When the body is moving, it is usually implemented through the cooperation of multiple muscle groups, and the posture information of human body can be detected by some wearable devices [15–18]. In this study, by detecting the sEMG signals of the upper limb, the motion posture of holding the steering wheel was identified, and the identified mode was converted into control commands to perform real-time control of virtual driving. The plantar pressure signals of subjects were collected by using the membrane pressure sensors, and the human gait was identified by combining the triaxial acceleration signal. The principle framework of wearable human posture detection is shown in Figure 1. Firstly, the original sEMG signals, triaxial acceleration signals, and plantar pressure signals were filtered. Secondly, the features of motion segment signals were extracted. Finally, the optimized SVM algorithm was used to identify the motion intention of human body.

### 2.1. Active Segment Detection and Feature Extraction of Upper Limb sEMG

In order to extract the motion information effectively, moving average window and threshold comparison are combined to detect active segment of the sEMG signal. The method is as follows:

(1) The sEMG signal sequence sEMG_*k*_(*i*) after the band-pass filtering is squared, and the instantaneous average energy sequence sEMG_*M*_(*i*) is defined. *i* is the current sEMG sequence label, that is,
  (1) $$\begin{array}{c} {\text{sEMG}}_{M}\left(i\right)={\left[{\text{sEMG}}_{k}\left(i\right)\right]}^{2}. \end{array}$$
(2) A moving window is selected with fixed window length *N*(*n* − 128), and the average energy sEMG_MA_(*i*) is calculated, that is,
  (2) $$\begin{array}{c} {\text{sEMG}}_{\text{MA}}\left(i\right)=\frac{1}{N}\overset{i+N}{\underset{j=i}{\sum }}{\text{sEMG}}_{M}. \end{array}$$
(3) The threshold *T* is set. If sEMG_MA_(*i*) ≥ *T* , all data in the window after time *t* are greater than the threshold *T*, and all data in the window before time *t* are less than the threshold *T*, then it is the starting point of the motion; otherwise, it is the ending point. In this study, 2% of the maximum energy of the sequence signal was selected as the threshold *T*[19].

The feature extraction is the key technique for the sEMG signal identification. Therefore, the selection of appropriate feature directly affects the subsequent classification results. In this study, the standard deviation and singular values of wavelet coefficients were selected as the features of pattern recognition [20, 21].

#### 2.1.1. Standard Deviation (SD)

(3) $$\begin{array}{c} \text{SD}=\sqrt{\frac{1}{N}\overset{N}{\underset{i=1}{\sum }}{\left(x_{i}-\bar{x}\right)}^{2}}, \end{array}$$

where *N* is the number of sampling points, *x*_*i*_ is the amplitude of sEMG signal at the *i* th sampling point, and $\bar{x}$ is the sample mean.

#### 2.1.2. Singular Value Decomposition (SVD)

The singular values of wavelet coefficients represent good stability and can fully reflect the information contained in the matrix. Let *A* ∈ *R*^*m∗n*^, and then there exists an orthogonal matrix *U*=[*u*_1_,…, *u*_*m*_] ∈ *R*^*m∗n*^, *V*=[*v*_1_,…, *v*_*m*_] ∈ *R*^*m∗n*^, such that

(4) $$\begin{array}{c} \;U^{T}\text{AV}=\text{diag}\left(\sigma_{1},\ldots ,\sigma_{\varphi }\right), \end{array}$$

where *p*=min(*m*, *n*),  *σ*_1_ ≥ *σ*_2_ ≥ ⋯≥*σ*_*φ*_ > 0, *σ*_*i*_,  (*i*=1, ⋯, *p*) is called the singular value of matrix *A*, that is, the positive square root of the eigenvalue *γ*_*i*_ of *AA*^*H*^ or *A*^*H*^*A*.

By decomposing the sEMG signal into level=3 ~ 5 layers, the level+1 subbands are obtained. Then, the singular value *σ*_*i*_ is achieved in each subband signal *S*_*i*_ by singular value decomposition. In this study, the singular value of each subband was used as the feature, that is, feature={*σ*_*i*_,  *i*=1,…, level+1}.

### 2.2. Gait Information Detection and Feature Extraction

The triaxial acceleration of the lower limb and plantar pressure signals were extracted. For time domain feature, acceleration mean $\bar{X}$, standard deviation *σ*, and variance *S*^2^ were extracted from three direction acceleration signals after preprocessing. For time-frequency domain feature, the wavelet energy spectrum was used.

The wavelet energy spectrum is based on the wavelet packet decomposition to extract multiscale spatial energy features. It calculates the energy in different decomposition scales and then arranges these energy values into the features according to the scale order, that is,

(5) $$\begin{array}{c} E\left(i,j\right)=\sum_{i=0}^{n-1}d{\left(i,j\right)}^{2}, \end{array}$$

where *d*(*i*, *j*) is the coefficient of wavelet packet transform, and *j* is the sequence number of low-frequency subspaces. In this study, the wavelet basis function db1 was selected for three-level decomposition. Eight low-frequency subspace acceleration signals were selected to extract wavelet packet energy.

The feature of plantar pressure signal extraction is the mean $\bar{F}$ of the difference between the forefoot pressure and the heel pressure, that is,

(6) $$\begin{array}{c} \bar{F}=\frac{1}{N}\left(\overset{N}{\underset{i=1}{\sum }}\left(F_{i}-f_{i}\right)\right), \end{array}$$

where *F*_*i*_ represents the forefoot pressure collected by the membrane pressure sensor, and *f*_*i*_ represents the heel pressure.

### 2.3. Optimized SVM Based on Genetic Algorithm

Compared with Bayes, K-nearest neighbor, decision tree, and other classification methods based on statistical pattern recognition, the SVM algorithm represents obvious advantages in solving small sample, nonlinear, and high-dimensional recognition problems [22, 23].

The principle of SVM algorithm means finding an optimal classification hyperplane to meet the classification requirements based on structural risk minimization, and its learning strategy is employed to maximize the interval, which is transformed into the solution of quadratic programming problem. For linearly inseparable data, it is firstly necessary to confirm the kernel function, and then the nonlinear mapping algorithm is used to transform the inseparable samples of low-dimensional features into high-dimensional features to make them linearly separable. The appropriate kernel function  *K*(*x*_*i*_, *x*) and parameter *C* are chosen. By constructing Lagrange dual function, the nonlinear SVM can be described as

(7) $$\begin{array}{c} \begin{array}{cc} \min_{\alpha } & \frac{1}{2}\overset{m}{\underset{i=1}{\sum }}\overset{m}{\underset{j=1}{\sum }}\alpha_{i}\alpha_{j}y_{i}y_{j}x_{i}^{T}x_{j}-\overset{m}{\underset{i=1}{\sum }}\alpha_{i},\\ \text{s.t.} & \;\overset{m}{\underset{i=1}{\sum }}\alpha_{i}y_{i}=0,0\ll \alpha_{i}\ll C,\;i=1,2,\ldots ,m, \end{array} \end{array}$$

where *C* is the penalty factor, and *α* is the Lagrange multiplier. The optimal solution of each coefficient is obtained. After the kernel function is confirmed, the optimal classification function is

(8) $$\begin{array}{c} f\left(x\right)=\mathrm{sgn}\left(\hat{\omega }\varphi \left(x\right)+\hat{b}\;\right)=\mathrm{sgn}\left[\overset{m}{\underset{i=1}{\sum }}\hat{\alpha_{i}}y_{i}K\left(x_{i},x\right)+\hat{b}\right]. \end{array}$$

The kernel functions used in the SVM algorithm include polynomial kernel function, Sigmoid kernel function, and radial basis function (RBF). In this study, the RBF was chosen, namely, *K*(*x*_*i*_, *x*)=exp(−*γx* · *x*_*i*_)^2^. Meanwhile, the genetic algorithm (GA) was used to optimize the parameters of kernel function.

The GA is a kind of quasinatural search algorithm based on Darwinian evolution theory. It can simulate the evolution of survival of the fittest in nature and map the problem-solving space to the genetic space. In order to optimize the SVM algorithm based on the GA, penalty factor *C* and RBF parameter *γ* need to be optimized. By selection, crossover, mutation, and other genetic operators, the population with good fitness is retained, and the optimal population is finally achieved by the iterative evolution. The flow chart of kernel function parameter optimization of the SVM based on the GA is shown in Figure 2.

## 3. Experimental Results

Twelve subjects were enrolled in the virtual driving control and gait experiment. The subjects consisted of six males and six females ranging in age from 21 to 27 years. All subjects did not have sprain and other injuries affecting motor function, as well as motor nerve diseases. The sEMG signals of upper limb were collected by DELSYS testing system, whose sensors used built-in electrodes with the spacing of 10 mm. All data between the electrodes and the receiver were transmitted by the wireless way. In the gait test, the subjects wore shoes with two membrane pressure sensors, and the triaxial acceleration acquisition device was placed at the ankle to collect the signals of five gait modes, including walking, waiting, going upstairs, going downstairs, and falling.

Some settings of control parameters used in this study are given in Table 1. In the process of GA optimization training, a 5-fold cross-validation was selected to obtain the optimal fitness. After 50 iterations, the optimal penalty factor *C*=5.0981 and kernel function parameter *γ*=1.0197 were calculated.

### 3.1. sEMG Identification Test

Each motion signal was collected by two channels.  Figure 3 shows three motion states of virtual vehicle, including left turn, stop, and right turn. The red circles in the figure represent the acquisition place of sEMG signals.

The effects of three motion states in the forearm muscles are different. Two groups of muscles, biceps brachii and extensor carpi ulnaris, are selected for the experiment. The time domain features of the left turn, stop, and right turn are shown in Table 2. Based on the results of standard deviation, it was found that the states of biceps brachii were more obvious in identifying three motions.

In order to further improve the identification accuracy, time-frequency feature fusion was performed. The standard deviation was selected for time domain feature, and wavelet coefficients were selected for frequency domain features. A set of low-frequency coefficients a3 and high-frequency coefficients d1, d2, and d3 could be obtained by three-level wavelet decomposition of the collected sEMG signals. The variance, maximum value, and singular values of the coefficients were calculated. It can be seen from Table 3 that the singular value features of wavelet coefficients are more obvious.

As can be seen from Figure 4, the combination of standard deviation and singular values of wavelet coefficients can achieve the highest identification accuracy through online recognition of the SVM algorithm. The identification accuracy for the left turn is 82%, that for the right turn is 92%, that for the stop is 98.7%, and the average identification accuracy of three motions is 90.90%.

Veer et al. applied neural network classifier to implement the classification of sEMG signals from upper arm muscles, and the best classification accuracy was 89.3% [24]. Zhang et al. recognized sEMG signals based on human motion intention, and the classification accuracy of upper limb signals based on SVM classifier was improved, ranging from 90.33% to 91.1% [25]. In comparison, our recognition results are better. Li et al. studied the quantitative relationship between sEMG signal features and upper limb joint angle, so as to identify the motion intention [26]. Shao et al. integrated the SVD feature to improve the classification accuracy effectively [27]. Tosin et al. also performed multiple feature analysis of sEMG signals from the upper limb [28]. These results show that multiple feature fusion can improve the classification accuracy.

It can be seen that real-time interaction with the virtual driving scene can be performed by detecting the sEMG signals of the upper limb and identifying the motion posture of holding the steering wheel in the virtual driving operation. Nacpil et al. also proposed a method to perform sEMG-controlled virtual car in a PC platform, which showed the feasibility for implementing a sEMG-machine interface that controlled the steering of the virtual car [29].

### 3.2. Gait Identification Test

Figure 5 shows acceleration and plantar pressure signals of five gait modes for walking, waiting, going upstairs, going downstairs, and falling.

After optimizing the parameters of the SVM, the identification accuracy comparisons are shown in Figure 6. The average gait identification accuracy based on single acceleration signals is 80.42%, and that based on plantar pressure signals is 69.28%. After fusing acceleration and plantar pressure signals, the average identification accuracy of the five gait modes is 90.48%, which is significantly higher than those based on single signal. Ai et al. combined wavelet coefficients and acceleration signal features, and based on SVM classifier, the classification accuracy of the five lower limb movements was increased by 8% [30], while our classification accuracy was increased by 12.5%.

## 4. Conclusion

In this study, the sEMG signal analysis and virtual driving technology were combined to study the effective feature extraction and classification identification method. Combined with the advantages of immersion, interest, and pertinence, the virtual driving control was performed by real motions. The biceps brachii muscle could distinguish three kinds of motions including left turn, stop, and right turn. The moving average window and threshold comparison were used to detect and segment the collected sEMG signals. The standard deviation and singular values of wavelet coefficients were extracted as the features. The SVM algorithm was used to perform real-time control of three virtual driving motions. The average identification accuracy was 90.90%.

The triaxial acceleration and plantar pressure signals for walking, waiting, going upstairs, going downstairs, and falling were collected, and the features of acceleration mean, standard deviation, variance, wavelet energy spectrum of acceleration signal,and mean of pressure difference between the forefoot and the heel were selected. By the optimized SVM, the average identification accuracy of five gait modes could reach 90.48%. The identification accuracy of fusion signal was significantly higher than that of the single signal.

The wearable human posture detection can be used for patients who need muscle rehabilitation training. It not only solves the problem of inconvenient operation for patients with motor dysfunction, but also has important practical significance for improving the rehabilitation training effect of patients.

## Figures and Tables

**Figure 1:** Principle framework of wearable human posture detection.

**Figure 2:** Flow chart of kernel function parameter optimization based on the GA.

**Figure 3:** Three motion states of virtual vehicle. (a) Left turn, (b) stop, (c) right turn.

**Figure 4:** Accuracy comparisons for three motion states.

**Figure 5:** Acceleration and plantar pressure signals.

**Figure 6:** Accuracy comparisons of five gait identification results.

**Table 1:** Parameters for the GA.

Parameter	Setting
Population size	50
Maximum generation	50
Gap probability	0.95
Crossover probability	0.8
Mutation probability	0.1
Kernel function	RBF

**Table 2:** Time domain features in different muscle positions.

Muscles	Features	Left turn	Stop	Right turn
Biceps brachii	Mean absolute value	67.2572 ± 12.2266	19.5647 ± 0.1265	21.3071 ± 12.2266
	Standard deviation	103.8934 ± 22.1665	5.3235 ± 1.2139	29.2781 ± 22.1665
	Variance	104.4871 ± 22.0447	20.2829 ± 0.3369	32.1099 ± 22.0447

Extensor carpi ulnaris	Mean absolute value	55.0021 ± 9.7912	19.5647 ± 0.1265	26.7749 ± 9.7912
	Standard deviation	88.8508 ± 16.1424	5.3235 ± 1.2139	43.4217 ± 16.1424
	Variance	88.8615 ± 16.1262	20.2829 ± 0.3369	43.4867 ± 16.1262

**Table 3:** Feature comparisons of wavelet coefficients for three motion states.

Features	Wavelet coefficients	Left turn	Stop	Right turn
Variance	a3	0.0007 ± 0.0004	5.6273e-06 ± 2.1938e-06	4.6795e-05 ± 3.9365e-05
	d3	0.0010 ± 0.0005	2.2806e-06 ± 1.1195e-06	8.2666e-05 ± 7.4132e-05

Maximum value	a3	118.7533 ± 48.8894	13.0637 ± 1.2329	23.5794 ± 19.2797
	d3	222.2225 ± 98.4360	6.9295 ± 2.5674	54.2183 ± 29.2419

Singular value	a3	1212.8528 ± 269.3678	560.9698 ± 12.5829	588.7500 ± 83.4251
	d3	1308.7037 ± 318.5597	41.6474 ± 10.4164	364.3723 ± 185.9567

## Data Availability

The ^∗^data used to support the findings of this study are available from the corresponding author upon request.

## References

[1] Farina D., Ning Jiang N., Rehbaum H. (2014). The extraction of neural information from the surface EMG for the control of upper-limb prostheses: emerging avenues and challenges. *IEEE Transactions on Neural Systems and Rehabilitation Engineering*.

[2] Ishii C. (2017). Control of an electric wheelchair based on EMG, EOG and EEG. *Journal of the Japan Society for Precision Engineering*.

[3] Fahreddin S., Cemal K., Berk D. (2017). Electromyogram (EMG) signal detection, classifiation of EMG signals and diagnosis of neuropathy muscle disease. *Procedia Computer Science*.

[4] Rincon A. L., Yamasaki H., Shimoda S. (2016). Design of a video game for rehabilitation using motion capture, EMG analysis and Virtual Reality. *International Conference on Electronics*.

[5] Powell M. A., Kaliki R. R., Thakor N. V. (2014). User training for pattern recognition-based myoelectric prostheses: improving phantom limb movement consistency and distinguishability. *IEEE Transactions on Neural Systems and Rehabilitation Engineering*.

[6] Sprager S., Juric M. (2015). Inertial sensor-based gait recognition: a review. *Sensors*.

[7] Cordoba R., Ferreiros J. (2016). Frequency features and GMM-UBM approach for gait-based person identification using smartphone inertial signals. *Pattern Recognition Letters*.

[8] Warren M. (1996). The effect of stimulus pulse duration on selectivity of neural stimulation. *IEEE Transactions on Biomedical Engineering*.

[9] Marcin D., Mariusz B. (2018). Recognition of a person wearing sport shoesor high heels through gait using two types of sensors. *Sensors*.

[10] Young S. C., Hojoon K., Doik K. (2018). Flexible piezoelectric sensor-based gait recognition. *Sensors*.

[11] Omid D., Mojtaba T., Raghvendar C. V. (2017). IMU-based gait recognition using convolutional neural networks and multi-sensor fusion. *Sensors*.

[12] Franchino P., Anana V. R., Deepak K. (2018). Wearable movement sensors for rehabilitation: a focused review of technological and clinical advances. *Innovations Influencing Physical Medicine and Rehabilitation*.

[13] Clayton R. P., Danilo R. P., Silke A. T. W., Christian H., Victor H. C. A., Joao P. P. (2019). A survey on computer- assisted Parkinson’s disease diagnosis. *Artificial Intelligence in Medicine*.

[14] Morales J., Akopian D. (2017). Physical activity recognition by smartphones a survey. *Biocybernetics and Biomedical Engineering*.

[15] Nackaerts E., Vervoort G., Heremans E., Smits-Engelsman B. C. M., Swinnen S. P., Nieuwboer A. (2013). Relearning of writing skills in Parkinson’s disease: a literature review on influential factors and optimal strategies. *Neuroscience & Biobehavioral Reviews*.

[16] Katzschmann R. K., Araki B., Rus D. (2018). Safe local navigation for visually impaired users with a time-of-flight and haptic feedback device. *IEEE Transactions on Neural Systems and Rehabilitation Engineering*.

[17] Ton C., Omar V. A., AftabTran A., Perla F., Bernstein M. J., Yang Y. (2018). LIDAR assist spatial sensing for the visually impaired and performance analysis. *IEEE Transactions on Neural Systems and Rehabilitation Engineering*.

[18] Kobsar D., Olson C., Paranjape R., Barden J. M. (2014). The validity of gait variability and fractal dynamics obtained from a single, body-fixed triaxial accelerometer. *Journal of Applied Biomechanics*.

[19] Li X., Zhou Z., Liu W., Ji M. (2019). Wireless sEMG-based identification in a virtual reality environment. *Microelectronics Reliability*.

[20] Gokgoz E., Subasi A. (2015). Comparison of decision tree algorithms for EMG signal classification using DWT. *Biomedical Signal Processing and Control*.

[21] Hariharan M., Fook C. Y., Sindhu R., Ilias B., Yaacob S. (2012). A comparative study of wavelet families for classification of wrist motions. *Computers & Electrical Engineering*.

[22] Quitadamo L. R., Cavrini F., Sbernini L. (2017). Support vector machines to detect physiological patterns for EEG and EMG-based human-computer interaction: a review. *Journal of Neural Engineering*.

[23] Sarkar J. A. M. (2014). Hidden Markov mined activity model for human activity recognition. *International Journal of Distributed Sensor Networks*.

[24] Veer K., Vig R. (2017). Analysis and recognition of operations using SEMG from upper arm muscles. *Expert Systems*.

[25] Zhang L., Liu G., Han B., Wang Z., Zhang T. (2019). sEMG based human motion intention recognition. *Journal of Robotics*.

[26] Li C., Zhou Y., Li Y. (2018). The signal processing and identification of upper limb motion based on sEMG. *Wireless Personal Communications*.

[27] Shao J., Niu Y., Xue C. (2020). Single-channel SEMG using wavelet deep belief networks for upper limb motion recognition. *International Journal of Industrial Ergonomics*.

[28] Tosin M. C., Cene V. H., Balbinot A. (2020). Statistical feature and channel selection for upper limb classification using sEMG signal processing. *Research on Biomedical Engineering*.

[29] Nacpil E. J., Zheng R., Kaizuka T., Nakano K. (2018). Implementation of a sEMG-machine interface for steering a virtual car in a driving simulator. *Advances in Intelligent Systems and Computing*.

[30] Ai Q., Zhang Y., Qi W., Liu Q., Chen a. K. (2017). Research on lower limb motion recognition based on fusion of sEMG and accelerometer signals. *Symmetry*.

